# Increasing Dietary Fat Elicits Similar Changes in Fat Oxidation and Markers of Muscle Oxidative Capacity in Lean and Obese Humans

**DOI:** 10.1371/journal.pone.0030164

**Published:** 2012-01-12

**Authors:** Audrey Bergouignan, Wendolyn S. Gozansky, Daniel W. Barry, Wayne Leitner, Paul S. MacLean, James O. Hill, Boris Draznin, Edward L. Melanson

**Affiliations:** 1 Center for Human Nutrition, School of Medicine, University of Colorado Denver, Denver, Colorado, United States of America; 2 Division of Geriatric Medicine, School of Medicine, University of Colorado Denver, Denver, Colorado, United States of America; 3 Division of Endocrinology, Metabolism, and Diabetes, School of Medicine, University of Colorado Denver, Denver, Colorado, United States of America; 4 Division of General Internal Medicine, School of Medicine, University of Colorado Denver, Denver, Colorado, United States of America; 5 Section of Nutrition, Department of Pediatrics, School of Medicine, University of Colorado Denver, Denver, Colorado, United States of America; Institut Pluridisciplinaire Hubert Curien, France

## Abstract

In lean humans, increasing dietary fat intake causes an increase in whole-body fat oxidation and changes in genes that regulate fat oxidation in skeletal muscle, but whether this occurs in obese humans is not known. We compared changes in whole-body fat oxidation and markers of muscle oxidative capacity differ in lean (LN) and obese (OB) adults exposed to a 2-day high-fat (HF) diet. Ten LN (BMI = 22.5±2.5 kg/m^2^, age = 30±8 yrs) and nine OB (BMI = 35.9±4.93 kg/m^2^, 38±5 yrs, Mean±SD) were studied in a room calorimeter for 24hr while consuming isocaloric low-fat (LF, 20% of energy) and HF (50% of energy) diets. A muscle biopsy was obtained the next morning following an overnight fast. 24h respiratory quotient (RQ) did not significantly differ between groups (LN: 0.91±0.01; OB: 0.92±0.01) during LF, and similarly decreased during HF in LN (0.86±0.01) and OB (0.85±0.01). The expression of pyruvate dehydrogenase kinase 4 (PDK4) and the fatty acid transporter CD36 increased in both LN and OB during HF. No other changes in mRNA or protein were observed. However, in both LN and OB, the amounts of acetylated peroxisome proliferator-activated receptor γ coactivator-1-α (PGC1-α) significantly decreased and phosphorylated 5-AMP-activated protein kinase (AMPK) significantly increased. In response to an isoenergetic increase in dietary fat, whole-body fat oxidation similarly increases in LN and OB, in association with a shift towards oxidative metabolism in skeletal muscle, suggesting that the ability to adapt to an acute increase in dietary fat is not impaired in obesity.

## Introduction

Although genetics is a contributing factor [1], the rapid increase in the prevalence of obesity suggests that environmental factors increase the risk of obesity in susceptible individuals. One such environmental factor may be a high intake of dietary fat [2], [3], [4]. Unlike carbohydrate and protein [5], [6], [7], when dietary fat intake increases, fat oxidation slowly increases over several days until oxidation matches intake [8], [9], which in absence of a compensatory increase in energy expenditure will result in an increase in fat mass [10]. Since low rates of fat oxidation are associated with gains in fat mass over time [11], [12], studying the effects of increased dietary fat intake on fat oxidation and its regulatory pathways may yield insight into susceptibility to weight gain.

It has been suggested that the ability to adapt to a high fat diet (HF) is impaired in obese individuals [13], [14] but few studies have directly compared lean and obese humans. Although studying changes in whole body fat oxidation provides some insight on the capacity to respond to changes in nutrient availability, studying changes at the molecular level in metabolically active tissues such as skeletal muscle will enhance the understanding of the pathophysiology of obesity. Studies in non-obese humans have demonstrated that increasing fat intake increases the expression, translation, and activity of several mediators of fat uptake and oxidation in skeletal muscle such as lipoprotein lipase (LPL) [15], the fatty acid transporter CD36 [16], and pyruvate dehydrogenase kinase 4 (PDK4) [16], [17], [18], [19], [20]. Collectively, these results suggest that in metabolically healthy individuals, increasing fat intake induces changes in skeletal muscle that increases fat oxidation and reduces carbohydrate oxidation. Skeletal muscle oxidative capacity is regulated by the complex interaction between 5-AMP-activated protein kinase (AMPK), silent mating type information regulation 2 homolog 1 (SIRT1) [21], [22], [23], and peroxisome proliferator-activated receptor γ coactivator-1-α (PGC1-α) [24], [25], [26]. AMPK and SIRT1 are intracellular fuel sensors that respond to changes in nutrient and energy availability [27]. PGC1- α is a nuclear encoded protein that is activated by AMPK and SIRT1 [28], and coactivates transcription factors and nuclear receptors that control cell function, including the expression of genes involved in fatty acid oxidation [25]. How increasing fat intake affects this network in skeletal muscle is not completely understood. Although studies in rodent models have shown increases in SIRT1, AMPK, and PGC1- α mRNA and protein in response to high fatty acid loads [29], [30], [31], [32], a study in lean humans reported a *decrease* in the mRNA of PGC1- α and other genes associated with oxidative capacity in response to an increase in dietary fat intake [33]. To our knowledge, only one study has compared the molecular adaptations to a HF diet in lean and obese humans [34]. In that study, the expression of PDK4 and PGC1- α increased in lean but decreased in the obese subjects, suggesting an impaired adaptation in the muscle of the obese subjects. The extent that these effects lead to changes in protein levels of these genes or in whole body substrate oxidation has not been investigated.

The purpose of this study was to test the hypothesis that obese, non-diabetic humans have an impaired ability to adapt to a HF diet. To do so, we compared changes in 24h fat oxidation and changes in gene expression, protein content, and post-transcriptional regulation of proteins regulating fat metabolism in muscle in lean and obese individuals in response to an increase in dietary fat intake.

## Methods

### Institutional Approval

The study was approved by the Colorado Multiple Institutional Review Board (COMIRB) and the Scientific Advisory Board of the Clinical Translation Research Center (CTRC) at the University of Colorado-Denver (UCD). Informed written consent was obtained from each subject. Subject recruitment began in January, 2007, and subjects were studied between February, 2007 and March, 2009.

### Subjects

Healthy lean (LN, body mass index (BMI)  = 19–25 kg/m^2^), and obese (OB, BMI  = 30–40 kg/m^2^) adults (20–45 years) were recruited for this study. Respondents were queried about their age, current and past body weight, physical activity patterns, and health history during an initial telephone screening. Inclusion criteria were self-reported weight stability (less than 5% change in body weight over the previous 6 months), a sedentary lifestyle (<1 exercise bout/week and sporting activities <1 hr/wk) and no history of prior obesity in lean subjects. Additional exclusion criteria for female volunteers were pregnancy or lactation, amenorrhea (absence of three or more consecutive menstrual cycles), self-reported abnormal menstrual cycle length (<26 days or >32 days), and post-menopausal status. Screening procedures confirmed that volunteers were healthy and non-diabetic [35]. Volunteers who passed the initial screening provided informed written consent, and were then invited to participate in a health history and physical examination. BMI was confirmed by measuring height and weight while wearing only socks, undergarments, and a hospital gown. After acceptance into the study, resting metabolic rate and body composition were measured, as described previously [35]. The characteristics of the 19 subjects included in this study are presented in Table 1. As expected, weight, BMI, and percent body fat were higher in OB than in LN (P<0.05).

**Table 1:** Subject characteristics.

		All subjects		Subjects with muscle biopsies	
	Lean		Obese	Lean	Obese
n	10		9	5	6
Sex	6F/4M		4F/5M	1F/4M	4F/2M
Age	30±8		37±7	31±10	38±7
BMI (kg/m2)	22.5±2.1		35.3±4.3*	22.9±2.5	35.1±4.1*
waist circumference (cm)	78.3±7.4		107.9±16.4*	82.7±7.0	111.0±14.5*
Weight (kg)	66.7±7.6		111.0±22.7*	71.2±6.5	106.1±17.1*
Fat-free mass (kg)	48.9±7.7		63.9±11.4*	54.1±7.6	62.2±9.6
Fat mass (kg)	17.6±4.6		42.2±8.9*	17.0±5.4	43.5±8.1*
% Fat mass (%)	26.6±6.5		39.5±3.3*	24.0±7.8	41.1±3.1*
Fasting insulin (mUI/l)	9.4±2.7		18.3±8.6*	11.0±1.7	18.7±9.2
Fasting glucose (mg/dl)	79.3±12.7		85.8±7.7	90.0±7.2	83.5±8.3
HOMA-IR	1.89±0.73		3.87±1.86*	2.45±0.46	3.81±1.87
Fasting cholesterol (mg/dl)	155.9±18.2		163.4±34.9	147.4±21.4	178.3±31.3
Fasting triglycerides (mg/dl)	88.7±25.1		142.9±77.7*	100.2±30.8	164.3±88.0

All values are mean±SD.

*P<0.05 versus Lean group.

### Study design

This study was conducted as part of a larger study of the effects of exercise (EX) and HF diets on substrate oxidation [35]. Subjects completed three trials, each separated by 1–3 weeks. The first trial served as the low fat control condition (LF), which was performed first to confirm that energy balance was achieved during the calorimeter stay. Subjects then performed either the EX or HF diet conditions in random order. Only data from the LF and HF conditions are presented here. Each condition lasted four days; subjects consumed a controlled outpatient diet on days 1–3 (to stabilize energy and macronutrient intake), and were studied in the room calorimeter on day 4. During the LF condition, subjects consumed the LF diet on days 1–4. During the HF diet condition, subjects consumed the LF diet for days 1–2, and then switched to a HF diet on days 3–4. Thus, the calorimeter measurements were obtained 24–48 hrs after the increase in dietary fat intake. We purposely chose this time frame based on our review of previous studies. Although complete adaptation to an isocaloric HF diet may take upwards of 7 days [8], a rapid and dramatic shift in substrate oxidation occurs within the first 24–48 hrs in both lean and obese subjects, as has been demonstrated in several studies [36], [37], [38]. Moreover, the magnitude to change in substrate oxidation is most pronounced within this first 24–48 hrs. Subjects were provided all meals during the four day trials. Subjects were instructed to maintain their typical sedentary lifestyle during the outpatient phase.

### Study diets

Study diets were prepared using individual food preferences. Prior to the study, subjects completed a survey indicating types of foods they liked and disliked. Meals consisted primarily of whole foods, and the increase in dietary fat content was achieved primarily by substituting lower fat items (e.g. low fat cheese, milk, and yogurt) with higher fat versions. The LF and HF diets were matched for energy and protein content, but varied in the amount of fat (20% and 50%, respectively) and carbohydrate (65% and 35%, respectively). The diets had a similar proportion of mono-, poly, and saturated fats (as a percentage of fat calories). The LF diet was comprised of 8–12% mono-unsaturated fat (as a percent of total calories), 3–5% polyunsaturated, and no more than 6% saturated fat. The HF diet was comprised of 20–30% mono-unsaturated fats, 8–12% polyunsaturated fats, and no more than 16% saturated fat. All diets were designed by a trained nutritionist using ProNutra software (Viocare Nic, Princeton, NJ). The energy content of the diets was estimated to maintain energy balance, as described previously [39]. Meals were packaged and taken with the subject. All food was required to be consumed, and no other food was permitted. Two optional food modules (200 kcal each) were provided in the event that the subject experienced hunger. To verify compliance to the diets, subjects were required to return the empty food containers to the study personnel.

### Calorimeter protocol

Subjects entered the calorimeter at 0800 hrs and exited at 0700 hrs the following day. Three bouts of bench-stepping exercise (3×20 minutes at 72 steps/min) were performed each day at 0830, 1350, and 1850 to mimic free-living physical activity. Subjects were free to move about the calorimeter during other times of the day, but primarily this time was spent in sedentary behavior (reading, writing, computer use, watching TV). Subjects were instructed to remain awake and not to nap or perform any exercise other than that prescribed by the protocol, and to go to bed at the same time during each calorimeter stay. Subjects recorded their time to bed, and all subjects reported going to bed prior to 2300 hrs. Meals were provided at 0900, 1315, and 1730 hrs, and a light snack was provided at 2000 hrs. The distribution of total daily energy intake was 30% at each meal and 10% in the evening snack. Venous blood samples were obtained at several time-points. Since continuous or frequent blood sampling is not practical in the room calorimeter, we selected time points to represent fasting (prior to entry, after exiting the calorimeter) and before and after meals. To obtain blood samples, subjects extended their arm through a leak-free port in the calorimeter wall. Subjects exited the room at 0700 the following morning, at which time a muscle biopsy was obtained.

### 24 h EE and substrate oxidation

Calorimeter data were extrapolated to 24h values, based on average minute values. 24h energy expenditure (EE) and total substrate oxidation were determined from oxygen consumption (VO_2_), carbon dioxide production (VCO_2_) and nitrogen excretion in the urines, as previously described [35].

### Blood analyses

Whole blood (2.5 mL) was added to a preservative (3.6 mg EDTA plus 2.4 mg glutathione in distilled water). Serum was separated after spinning and stored at −80°C until analyzed. Fasting samples were assayed for glucose, insulin, triglycerides (TG), and FFA. All the other samples collected during the test were assayed for FFA and TG. Glucose concentrations were determined using the hexokinase method (Roche Indianapolis, IN)). Insulin concentrations were measured using standard, double antibody radioimmunoassay (Diagnostic Systems Laboratory, Webster, CT). FFA (Wako Chemical, Richmond, VA) and TG concentrations (Sigma Diagnostics, St. Louis, MO) were determined using enzymatic assays.

### Skeletal muscle biopsy

Muscle biopsies were obtained upon exiting the calorimeter on day 5. Subjects were fasted overnight prior to the biopsy. Subcutaneous tissue overlying the *vastus lateralis* muscle was infiltrated with 1% lidocaine. A small incision was made with a scalpel down through the level of the fascia. A Bergstrom side-cut biopsy needle with suction was used to remove approximately 0.25g of skeletal muscle tissue. Tissue samples were frozen immediately using the “freeze clamp” method. The biopsy samples were stored at −80°C until analyzed.

### Gene expression

After total RNA extraction, the relative expression levels of AMPKα2, CD36, cytochrome oxidase 4 (COX4), a marker of electron transport activity, PDK4, PGC1-α, LPL, SIRT1 were analyzed and quantified using the Experion System (Bio-Rad, Hercules, CA). Reverse transcription was performed using 250 ng total RNA with iScript cDNA synthesis kit (Bio-Rad). Quantitative PCR was performed using primer sets for genes of interest and two reference genes and iQ SYBR Supermix (Bio-Rad) following manufacturer's protocol. Reactions were run in duplicate on an iQ5 Real-Time PCR Detection System (Bio-Rad) along with a no-template control per gene. RNA expression data were normalized to levels of reference gene RPL13A and UBC using the comparative threshold cycle method. To demonstrate that efficiencies of target and reference genes are approximately equal, validation experiments were performed.

### Immunoblotting

The total amounts of AMPK, PGC1-α, and SIRT1 as well as phospho-AMPK and acetylated PGC-1α were determined by immunoblotting with the corresponding specific antibodies. Four hundred mcg of protein lysate were used to immunoprecipitate AMPK, PGC1-α, and SIRT1. PGC1- α lysine acetylation was analyzed by immunoprecipitation of PGC1- α followed by Western blot using acetyl-lysine antibodies (Cell Signaling Technologies, Danvers, MA, USA) as previously described [40]. Bovine serum albumin (BSA) and the protease inhibitors aprotinin and leupeptin were purchased from Boehringer Mannheim (Indianapolis, IN, USA). Protein Agarose beads, PGC1-α polyclonal antibody, AMPKα1/2 monocloanal antibody (#sc74461) and phospho-AMPK –Thr 172 antibodies as well as SIRT1 polyclonal antibody were purchased from Santa Cruz Biotechnology (Santa Cruz, CA, USA, and anti-mouse and anti-rabbit HRP labeled antibodies were from Amersham (Piscataway, NJ,). Electrophoretic gels, supplies and kits were obtaeind from BioRad Laboratories (Hercules, CA, USA).and GE Healthcare Bio Science/Amersham Biosciences (Piscataway, NJ, USA).

### Statistical Analysis

Statistical analyses were carried out using Graphpad Prism (Version 5.03, La Jolla, CA). To determine the effect of HF diet on 24 h substrate oxidation, substrate balance, and FFA and TG AUC, analyses used repeated measures ANOVA to account for repeated measurements on subjects during two conditions (LF diet versus HF diet) with group (LN versus OB) as main effect. For significant interactions, Tukey's post-hoc tests were performed to determine within group differences between conditions. If the interaction terms were non-significant, then the main effects of group and condition were evaluated. The effects of study diets on molecular adaptations at muscle level were also analyzed using repeated measures ANOVA. Significance for all tests was set at P = 0.05. Data are presented as Mean±SEM unless otherwise specified.

## Results

### Energy expenditure and energy balance

Absolute EE was significantly higher in OB compared to LN, but when expressed relative to FFM, there were no differences between groups (Table 2). 24 h EE did not differ between the LF and HF conditions in either LN or OB. Mean energy balance for each group was close to zero (<±85 kcal/day for each group and condition; Table 2), and did not differ between groups or conditions.

**Table 2:** Room calorimeter results (mean±SE).

		Lean (LN)			Obese (OB)				
		N = 10			N = 9			ANOVA P-value	
	LF		HF	LF		HF	Group	Condition	Interaction
*24 h Energy expenditure*									
*kcal/day* 1	2217±83		2161±88	3180±180		3133±180	<0.0001	*ns*	*ns*
*kcal/kg FFM/day*	45.7±1.2		46.6±0.8	44.5±1.2		45.9±0.8	*ns*	*ns*	*ns*
*Energy balance (kcal/day)*	42±41		84±48	−50±40		−33±75	*ns*	*ns*	*ns*
*Physical Activity Level (PAL)* 4	1.61±0.05		1.56 ±0.08	1.57±0.08		1.55±0.06	*ns*	*ns*	*ns*
*24 h RQ* 2	0.90±0.01		0.84±0.01	0.90±0.01		0.83±0.01	*ns*	<0.0001	*ns*
*Protein oxidation (g)* 1	72±6		77±8	101±9		105±6	<0.05	*ns*	*ns*
*Carbohydrate oxidation (g)* 1,2	344±24		256±20	507±53		320±40	<0.05	<0.0001	*ns*
*Fat oxidation (g)* 1,3	49±9		92±10	67±10		140±15	<0.05	<0.0001	*ns*

1 OB > LN.

2 LF > HF.

3 LF < HF.

4 PAL  = 24 h EE/resting metabolic rate.

RQ = respiratory quotient.

FFM = fat free mass.

FM = fat free mass.

### Twenty four hour substrate oxidation and balance

During LF diet, 24 h RQ did not significantly differ between groups (Table 2). After two days on the HF diet, twenty-four hour RQ was significantly reduced in both groups, but not different between LN (0.84±0.01) and OB (0.83±0.01). Absolute protein, carbohydrate and fat oxidation (g/day) were higher in OB than in LN (Table 2), but there was no between-group differences when expressed relative to FFM (g/kg FFM/24 h) (Figure 1). Twenty four hour protein oxidation did not differ on the LF and HF diets. However, 24 h fat carbohydrate oxidation was significantly lower and 24 h fat oxidation was significantly higher during HF (P<0.001) in both groups (Table 2, Figure 1). Twenty four hour protein balance (Figure 2) was slightly positive and did not differ on the LF and HF diets. In both groups, 24 h carbohydrate balance (Figure 2) was significantly lower (−88±20, and −187±50 g/day in LN, and OB, respectively) and 24 h fat balance (Figure 2) was significantly higher (+43±6, and +34±17 g/day in LN and OB, respectively) during HF compared to LF. The change in fat balance between LF and HF was not significantly different between LN and OB (P = 0.65, 95% CI  = −48.3 to +31.1 g/day).

**Figure 1:** Mean (± SE) Protein (Top), carbohydrate (Middle), and fat (Bottom) oxidation (g/kg FFM/day) measured using room calorimetry during LF (black bars) and HF (grey bars) in LN (N = 10) and OB (N = 9). * LF significantly different from HF (P<0.05).

**Figure 2:** Mean (± SE) 24 h (g/day) protein (Top), carbohydrate (Middle), and fat (Bottom) balance measured using room calorimetry during LF (black bars) and HF (grey bars) in LN (N = 10) and OB (N = 9). * LF significantly different from HF (P<0.05).

### Twenty four hour plasma FFA and triglycerides kinetics

To assess the overall effect of diet and obesity on FFA and TG concentrations, we calculated the area under the curve (AUC) of FFA and TG concentrations over 24hr (Figure 3). FFA AUC was significantly higher during HF in both LN and OB. The significant interaction (P = 0.04) suggests that the increase was greater in OB than LN. Although post-hoc analyses of the 24 h FFA profiles indicated some differences in FFA between LN and OB at different time points, the magnitude of these differences were small. TG AUC was significantly lower during HF in both LN and OB (P = 0.003), but not different between LN and OB (P = 0.07), Post-hoc analysis of the 24 h TG profiles indicated some differences in TG between LN and OB, particularly during the post-prandial period during the HF diet.

**Figure 3:** Plasma FFA (± SE; Left) and triglycerides (± SE; Right) during LF (Top) and HF (Middle) diets in LN (N = 10; dashed line), and OB (N = 9; solid line). 24 h FFA and triglycerides areas under the curve (AUC) are presented in the bottom graphs.

### Muscle gene expression

An insufficient quantity of muscle was obtained from the biopsy of several subjects; thus, the muscle analyses are based on samples obtained in five LN (1 female, 4 males) and six OB (4 females, 2 males) subjects. There were no differences in expression of AMPK, COX4, LPL, PGC1-α and SIRT1 in LN and OB. However, mRNA CD36 and PDK4 levels were higher in OB than in LN (P<0.01 for both). Increasing dietary fat intake did not change the expression of AMPK, COX4, LPL, PGC1-α or SIRT1 in either group (Table 3). However, increasing dietary fat intake significantly increased the expression of CD36 and PDK4 in both LN and OB. The increase in PDK4 mRNA was however more pronounced in OB than in LN subjects (P for interaction <0.01).

**Table 3:** mRNA results (au, mean±SE).

	Lean (LN)		Obese (OB)				
	N = 5		N = 6			ANOVA P-value	
	LF	HF	LF	HF	Group	Condition	Interaction
*AMPK*	0.75±0.06	0.81±0.08	0.67±0.05	0.77±0.05	*ns*	*ns*	*ns*
*CD36* 1,3	0.56±0.05	0.68±0.10	0.80±0.08	1.14±0.08	<0.01	<0.05	*ns*
*COX4*	0.06±0.01	0.07±0.01	0.06±0.01	0.06±0.01	*ns*	*ns*	*ns*
*LPL*	0.28±0.12	0.28±0.08	0.24±0.06	0.36±0.09	*ns*	*ns*	*ns*
*PDK4*	0.16±0.04	0.23±0.03	0.31±0.06	0.93±0.14	<0.01	<0.01	<0.01
*PGC1a*	0.66±0.08	0.57±0.09	0.54±0.04	0.62±0.04	*ns*	*ns*	*ns*
*SIRT1*	0.06±±0.01	0.08±0.01	0.06±0.01	0.08±0.01	*ns*	*ns*	*ns*

1 OB > LN.

2 LF > HF.

3 LF < HF.

### Muscle protein content and post-transcriptional regulation

The amount of SIRT1 protein in skeletal muscle did not differ between the HF or LF dietary conditions in both groups (data not shown). However, the significantly lower amount of acetylated PGC1-α during the HF diet (P<0.001, Figure 4, Bottom) coupled with no change in total PGC1-α protein (Figure 4, Top) suggests that the deacetylating activity of SIRT1 was markedly enhanced by the HF diet. Although the total amount of AMPK was not affected by the diet (Figure 5, Top), the HF diet significantly increased the phosphorylation of AMPK in both LN and OB (Figure 5, Bottom).

**Figure 4:** Mean (± SE) total (Top) and acetylated (Bottom) PGC1α protein (Bottom) during LF (black bars) and HF (grey bars) in LN (N = 5) and OB (N = 6). Representative blots are show above the graphs. * LF significantly different from HF (P<0.05).

**Figure 5:** Mean (± SE) total (Top) and phosphorylated (Bottom) AMPK protein during LF (black bars) and HF (grey bars) in LN (N = 5) and OB (N = 6). Representative blots are show above the graphs. * LF significantly different from HF (P<0.05).

## Discussion

Several studies have examined the effects of obesity on the ability to adapt to a HF diet [14], [36], [37], but few have actually compared obese and lean subjects. Two of these studies reported that when overfed a HF diet (resulting in positive energy balance), obese subjects had an impaired ability to increase fat oxidation [13], [14]. In the current study, although an isocaloric increase in dietary fat intake from 20% to 50% resulted in positive 24h fat balance in both LN and OB, the change in carbohydrate and fat oxidation and thus, the resulting fat balance, were similar. Moreover, changes in markers of skeletal muscle oxidative capacity were remarkably similar. Although no changes in PGC1-α, SIRT1, or AMPK mRNA or protein were observed, the amount of de-acetylated PGC1-α and pAMPK were increased in both LN and OB indicating an increase in the activity of both SIRT1 and AMPK respectively. The fact that 24hr fat oxidation and muscle oxidative capacity were not different in LN and OB groups in response to HF suggests that uptake by skeletal muscle was similar in LN and OB. Collectively, these results suggest that the ability to increase fat oxidation in response to an acute isocaloric increase in dietary fat intake is preserved in obese, non-diabetic humans at both the whole body and skeletal muscle level.

Although the observed increase in whole body fat oxidation is consistent with previous studies in humans [8], [9], [36], [41] the novel finding of the current study is that in obese, the ability to adapt to the increase in dietary fat intake is preserved, at least during isocaloric conditions. We also present novel findings regarding the effects on important cellular signaling molecules that regulate fat oxidation in skeletal muscle. An increase in dietary fat intake from 20% to 50% of total calories for two days induced significant changes in SIRT1 and AMPK activity, without changing the expression or translation of these proteins. There were also no changes in PGC1-α mRNA or protein. However, PGC1-α activity may be largely determined by post-translational modifications [28], [30], [40], as indicated by the change in acetylated PGC1-α observed in the current study. These results suggest that in humans, increasing fat intake for two days leads to changes in skeletal muscle that would be expected to increase oxidative capacity. These findings are consistent with studies in mice that have shown that raising serum FFA by feeding them HF diets [32] or combining HF diets with daily heparin injections [31] leads to a gradual increase in skeletal muscle PGC1-α protein and mitochondrial proteins over several weeks, suggesting that oxidative capacity is increased. It is likely that the relatively short exposure to the HF diet in the current study was not sufficient to induce changes in mRNA or protein of PGC1-α or SIRT1, as seen in the longer studies in mice.

Changes in FFA and TG in response to the HF diets were similar in LN and OB, i.e. FFA increased and TG decreased. The decrease in TG during HF diet is likely due to a decrease in carbohydrate availability, as has been previously been reported [42], [43], [44]. Although a significant difference in FFA AUC was observed, the magnitude of differences between LN and OB on both the LF and HF diets was small. We would contend that the physiological significance of such small differences is dubious. It is possible that these small differences were due to the study design, i.e., isocaloric LF and HF diets, and that larger differences would have been observed under conditions of energy surplus. Nonetheless, we concede that the small differences in the current study may conceal some underlying differences in FFA trafficking. It is possible that the higher TG concentrations in OB than LN, particularly during the post-prandial period, is related to the slightly higher plasma FFA concentrations in OB, since FFA is the main source for VLDL-TG synthesis [45]. Our findings that circulating FFA concentrations are slightly elevated in obese individuals is consistent with the observation by Karpe et al. [46] that although lipolysis and FFA delivery under fasting conditions is downregulated in obesity, an elevation in fasting FFA is observed in some obese individuals. In these individuals, it is likely that delivery of FFA to non-adipose tissue is increased. However, how lipolysis and FFA delivery during HF feeding is regulated in obese individuals during HF feeding has not been studied, to our knowledge. In our study, given that whole body fat oxidation did not differ in LN and OB during either diet condition, and that skeletal muscle is the primary tissue where fat is oxidized, it is possible that FFA delivery to other tissues (e.g. adipose tissue, liver) was increased in OB subjects. However without kinetic measurements, it is not possible to determine if differences in lipid trafficking contributed to these small differences in circulating FFA and TG.

The effect of increasing fat intake on molecular markers of fat oxidation in human skeletal muscle has not been well studied, and results from previous studies have been equivocal. In lean humans, increasing fat intake from 35% to 50% of total calories for three days induced a decrease in PGC1-α mRNA and other genes associated with oxidative capacity [33]. In a more recent study, exposure to a high fat diet (65%) for five days increased PGC1-α mRNA in lean but not obese subjects [34]. Possible reasons that may have contributed to different results (with regards to PGC1-α mRNA) of the current study and previous studies may include different levels of fat intake during the control and HF diet conditions and different length of exposure to the HF diets. It is also possible that differences in the types of fat (mono-, poly, and saturated) could contribute to differences between studies, but prior studies have not reported the distribution of fat calories in the experimental diets. It is also noteworthy that in contrast to our obese subjects, Boyle et al. [34] studied morbidly obese individuals (BMI>35 kg/m^2^). This raises the possibility that the ability to adapt to a HF diet may depend upon the level of excess adiposity. This remains an area for future investigation.

It has been previously shown that caloric restriction activates both AMPK and SIRT1 as an adaptive mechanism to increase ATP production from fat oxidation [47], [48], [49], [50]. Although the specific nutrient signals which activate the AMPK/SIRT1/PGC1-α pathways are not known, it has been speculated that fluctuations in nutrient supply may serve to synchronize this metabolic networks [51]. In line with this hypothesis, the results of the current study suggest that either a decreased availability of dietary carbohydrate or an excess availability of dietary fat may be one of the sensors that activate the AMPK/SIRT1/PGC1-α network. We could not, however, determine the specific intracellular signals that activated this network. Both SIRT1 and AMPK are activated by nutrient deprivation [51], [52]. AMPK is activated by increases in cellular AMP content, resulting in phosphorylation and activation of PGC-1α [53]. SIRT1 is activated by an increase in the cellular NAD^+^/NADH ratio, resulting in deacetylation and activation of PGC1-α [51], [54]. However, we cannot rule out the possibility that activation occurred via other pathways. For example, it was recently shown that a HF diet induced increases in NAD^+^ in liver and white adipose tissue, but not muscle [55], suggesting that NAD^+^ activation of SIRT1 may be tissue specific. Additionally, a recent study in humans demonstrated SIRT1 activity is not required for exercise-induced deacetylation of PGC1-α in muscle; deacetylation was induced via a novel acetyltransferase, general control of amino-acid synthesis-5 [56]. Results of these studies suggest that activation of PGC1-α activity in muscle is regulated on multiple levels that are not completely understood at the present time.

The activation of this network may have contributed to increase PDK4 gene expression [57], which plays a critical role in the partitioning of substrate toward either lipid or carbohydrate oxidation [58]. Although we were unable to assess PDK4 protein levels, it has been previously shown that HF diet simultaneously increases PDK4 mRNA and protein levels in lean subjects [16], [19]. Furthermore, although the increase in mRNA PDK4 in response to a HF diet is in accordance with several previous reports in lean subjects [17], [20], [34], it is the opposite of what Boyle et al [34] observed in morbidly obese individuals.

The strengths of this study include carefully targeted levels of energy balance, and the combined approach of measuring changes on the whole-body and molecular level. There are several limitations. Although we purposely studied subjects in energy balance, differences between groups may be more apparent during other conditions such as overfeeding, as has been previously demonstrated in lean vs. obese men [13]. Overfeeding appears to be necessary for the HF diet induced increase in energy expenditure and fat oxidation that occurs in obesity-resistant, but not obesity-prone, rats [59], [60]. We also studied subjects under controlled physical activity levels. It is well known that exercise increases fat oxidation, and that a more complete adaptation to an increase in dietary fat intake occurred when subjects are studied during high vs. low levels of physical activity (PAL = 1.8 vs. 1.4) [9]. The level of physical activity (PAL = 1.6) similar between groups may have impaired our ability to detect differences between lean and obese and studies with different levels of activity during the day of test may be warranted. Additionally, although the number of subjects in each group is similar or larger than previously published studies [9], [36], [37], [38], [41], [61], [62], we lacked sufficient statistical power to determine the effects of sex. Moreover, adequate muscle samples were available on only a subset of subjects, and the distribution of males and female samples differed in the LN and OB groups. However, given the robust and equal response in PGC1-α and pAMPK in both groups, it is unlikely that the sex distribution affected our results. We also lacked adequate samples to perform analyses of downstream or upstream markers of PGC1-α and SIRT1 activity such as changes in acetyl CoA carboxylase and NAD/NADH ratio, respectively. Finally, the length of the dietary intervention was very short. The changes induced by long-term exposure to excess dietary fat remain unknown. Performing such studies would enhance our knowledge of the mechanisms by which skeletal muscle regulates fatty acid oxidation, and would contribute to our understanding of the association between the pathophysiology of metabolic diseases.

In summary, results of this study demonstrate that increasing dietary fat intake increases whole-body fat oxidation, and this is accompanied by changes in skeletal muscle that reflect a shift towards oxidative metabolism. The response is similar in lean and obese individuals, suggesting that the ability to adapt to an acute increase in dietary fat is not impaired in obesity. We cannot rule out, however, that differences may have existed in the OB subjects prior to them becoming obese, and this is what contributed to the development of obesity in the first place. At the molecular level, substantial increases in the activity of SIRT1 and AMPK were observed, without changes in the message or protein. Thus, our data suggest that changes in skeletal muscle oxidative capacity cannot be inferred from changes in mRNA or protein expression. Despite these changes, fat balance was more positive during HF than LF in both groups, suggesting that HF diets will promote an increase in fat mass independent of energy intake under sedentary conditions. The results of the current study and those of Smith et al. [9] demonstrate that the best way to prevent against excess fat gain is to maintain daily physical activity and refrain from excessive consumption of dietary fat.
